The article "Mitochondrial aldehyde dehydrogenase (ALDH2) protects against streptozotocin-induced diabetic cardiomyopathy: role of GSK3β and mitochondrial function" was retracted in 2022. Reasons: duplicated images; concerns about the data.

# Mitochondrial aldehyde dehydrogenase (ALDH2) protects against streptozotocin-induced diabetic cardiomyopathy: role of GSK3β and mitochondrial function

**DOI:** 10.1186/1741-7015-10-40

**Published:** 2012-04-23

**Authors:** Yingmei Zhang, Sara A Babcock, Nan Hu, Jacalyn R Maris, Haichang Wang, Jun Ren

**Affiliations:** 1 Department of Cardiology, Xijing Hospital, Fourth Military Medical University, Xi'an, 710032, China; 2 Center for Cardiovascular Research and Alternative Medicine, University of Wyoming College of Health Sciences, Laramie, WY 82071, USA

**Keywords:** ALDH2, cardiac contraction, diabetes, GSK3β, mitochondrial function

## Abstract

**Background:**

Mitochondrial aldehyde dehydrogenase (ALDH2) displays some promise in the protection against cardiovascular diseases although its role in diabetes has not been elucidated.

**Methods:**

This study was designed to evaluate the impact of ALDH2 on streptozotocin-induced diabetic cardiomyopathy. Friendly virus B(FVB) and ALDH2 transgenic mice were treated with streptozotocin (intraperitoneal injection of 200 mg/kg) to induce diabetes.

**Results:**

Echocardiographic evaluation revealed reduced fractional shortening, increased end-systolic and -diastolic diameter, and decreased wall thickness in streptozotocin-treated FVB mice. Streptozotocin led to a reduced respiratory exchange ratio; myocardial apoptosis and mitochondrial damage; cardiomyocyte contractile and intracellular Ca^2+ ^defects, including depressed peak shortening and maximal velocity of shortening and relengthening; prolonged duration of shortening and relengthening; and dampened intracellular Ca^2+ ^rise and clearance. Western blot analysis revealed disrupted phosphorylation of Akt, glycogen synthase kinase-3β and Foxo3a (but not mammalian target of rapamycin), elevated PTEN phosphorylation and downregulated expression of mitochondrial proteins, peroxisome proliferator-activated receptor γ coactivator 1α and UCP-2. Intriguingly, ALDH2 attenuated or ablated streptozotocin-induced echocardiographic, mitochondrial, apoptotic and myocardial contractile and intracellular Ca^2+ ^anomalies as well as changes in the phosphorylation of Akt, glycogen synthase kinase-3β, Foxo3a and phosphatase and tensin homologue on chromosome ten, despite persistent hyperglycemia and a low respiratory exchange ratio. *In vitro *data revealed that the ALDH2 activator Alda-1 and glycogen synthase kinase-3β inhibition protected against high glucose-induced mitochondrial and mechanical anomalies, the effect of which was cancelled by mitochondrial uncoupling.

**Conclusions:**

In summary, our data revealed that ALDH2 acted against diabetes-induced cardiac contractile and intracellular Ca^2+ ^dysregulation, possibly through regulation of apoptosis, glycogen synthase kinase-3β activation and mitochondrial function independent of the global metabolic profile.

## Background

The mitochondrial isoform of aldehyde dehydrogenase (ALDH2) has been shown to play a pivotal role in the metabolism of acetaldehyde and other toxic aldehydes [1-4]. Ample evidence from our laboratory as well as others has revealed a rather singular role for ALDH2 in cardioprotection against ischemic injury, arrhythmias and alcoholism [2,3,5-7]. However, the role of ALDH2 in myopathic anomalies associated with metabolic disorders, including diabetes mellitus, has not been elucidated. The prevalence of diabetes and associated heart diseases has been steadily increasing, particularly in Asian countries, with approximately 50% of populations carrying one copy of the mutant ALDH2 gene [4,8-11]. A plethora of studies have depicted significant contribution from genetic variants, such as peroxisome proliferator-activated receptors (PPARs), in the predisposition of diabetes [12]; however, very few have examined the role of ALDH2 in the onset and progression of diabetes and its complications. Recent evidence revealed that ALDH2 polymorphism is closely associated with an increased risk of diabetes [11] while experimental findings showed reduced ALDH2 expression and activity associated with oxidative stress and cardiac dysfunction in diabetes [13]. These observations are somewhat consistent with the notion that inactive ALDH2 promotes hyperglycemia [9], while genotypes of ALDH2 can modify diabetes risk irrespective of alcohol intake [14]. To this end, this study was designed using a unique murine model to examine the impact of ALDH2 overexpression in the pathogenesis of diabetic cardiomyopathy and the underlying cellular mechanism(s) involved. Recent evidence from our group has revealed a pivotal role for the essential survival factor Akt and its downstream signaling molecules, including glycogen synthase kinase-3β (GSK3β), PPAR (mTOR) and the forkhead transcriptional factor in ALDH2, in cardioprotection against alcoholism and ischemia-reperfusion [3,7,15]. To better elucidate the interplay between these signaling cascades and mitochondrial function in diabetes and/or ALDH2-induced cardiac responses, we scrutinized apoptosis and mitochondrial integrity, including mitochondrial membrane potential, as well as cell signaling of Akt, GSK3β, mTOR and Foxo3a in wild-type FVB and ALDH2 transgenic mice with or without the induction of experimental diabetes. Given that Akt signaling is under the negative control of phosphatase and tensin homologue on chromosome ten (PTEN) in a wide variety of disease conditions, including myocardial hypertrophy, heart failure and preconditioning [16], we monitored pan protein expression and phosphorylation of PTEN. To evaluate if ALDH2 affects myocardial morphometric and functional anomalies in diabetes through any potential effect secondary to global metabolic alterations, we scrutinized whole body metabolism, including the respiratory exchange ratio (RER), and total physical activity as well as plasma levels of free fatty acid, insulin and glucose (fasting and postprandial) in control and diabetic mice.

## Methods

### Experimental animals, experimental diabetes and ALDH2 activity

All animal procedures were approved by our Institutional Animal Care and Use Committee at the University of Wyoming (Laramie, WY, USA). Production of ALDH2 transgenic mice using the chicken β-actin promoter was as described previously [5]. All mice were housed in a temperature-controlled room under a 12 hour light-12 hour dark circadian cycle with access to water and food *ad libitum*. Five-month-old male FVB (used as wild-type) and ALDH2 transgenic mice received intraperitoneal injections of streptozotocin (STZ, 200 mg/kg). All mice were maintained for four weeks with free access to standard laboratory chow and tap water before their blood glucose levels were monitored. Mice with fasting blood glucose levels > 13 mM were deemed diabetic [17].

ALDH2 activity was measured in 33 mM sodium pyrophosphate containing 0.8 mM NAD^+^, 15 μM propionaldehyde and 0.1 mL protein extract. Propionaldehyde, the substrate of ALDH2, was oxidized in propionic acid, while NAD^+ ^was reduced to NADH to estimate ALDH2 activity. NADH was determined by spectrophotometric absorbance at 340 nm. ALDH2 activity was expressed as nanomoles NADH per minute per milligram of protein [18].

### Serum free fatty acid, plasma insulin and blood glucose levels

Plasma free fatty acids were measured three hours after mice were denied access to food using a Free Fatty Acid Assay Kit (Cayman Chemical, MI, USA). In brief, mouse blood samples were centrifuged at 2000 × g for 15 minutes at 4°C. An excitation wavelength of 530 nm and an emission wavelength of 590 nm were used to detect the quantity of free fatty acids. Plasma insulin levels were measured using a mouse insulin ELISA kit from Diagnostic System Laboratory (Webster, TX, USA). Fasting (overnight) and postprandial (two hours after re-feeding following the overnight fasting) blood glucose levels were determined using a glucometer (Accu-ChekII, model 792, Boehringer Mannheim Diagnostics, Indianapolis, IN, USA) [17].

### Metabolic measurement

Indirect calorimetry and total physical activity were measured in light (10 a.m.) and dark (10 p.m.) phases using the Comprehensive Laboratory Animal Monitoring System (Oxymax/CLAMS; Columbus Instruments, Columbus, OH, USA). Volume of oxygen intake (VO_2_), volume of Carbon Dioxide exhaled (VCO_2_), the RER (VCO_2_/VO_2_) and physical activity were measured. All the parameters were measured every 10 minutes for six hours during daytime and six hours during nighttime. Result recorded in the first and last half hour was not be used. For simplicity, only the RER is presented without displaying original data from VO_2 _and VCO_2 _[19].

### Echocardiographic assessment

Cardiac geometry and function were evaluated in anesthetized mice using a two-dimensional guided M-mode echocardiography (Sonos 5500; Phillips Medical System, Andover, MA, USA) equipped with a 15-6 MHz linear transducer. Left ventricular (LV) wall thickness and diastolic and systolic dimensions were recorded from the M-mode images. Fractional shortening was calculated from end-diastolic diameter (EDD) and end-systolic diameter (ESD) using the equation:

(EDD-ESD)/EDD×0.01

Estimated echocardiographic LV mass was calculated as:

[(LVEDD+septal wall thickness+posterior wall thickness)3-LVEDD3]×1.055

where 1.055 (in mg/mm^3^) represents the density of the myocardium. Heart rate was calculated from 20 consecutive cardiac cycles [20].

### Isolation of murine cardiomyocytes

After intraperitoneal administration of a sedative (ketamine 80 mg/kg and xylazine 12 mg/kg), the hearts were removed and digested for 20 minutes with Liberase Blendzyme 4 (Hoffmann-La Roche Inc., Indianapolis, IN, USA). Cardiomyocyte yield was approximately 75% and was not affected by STZ treatment or ALDH2 overexpression. Only rod-shaped myocytes with clear edges were selected for the mechanical study [21].

For the *in vitro *study, cardiomyocytes from control FVB mice were exposed to high extracellular glucose (25.5 mM) [22] in the absence or presence of the ALDH2 activator Alda-1 (20 μM), the mitochondrial uncoupler carbonyl cyanide 4-trifluoromethoxyphenylhydrazone (FCCP, 1 μM) or the GSK3β inhibitor SB216763 (10 μM) [23,24] for 12 hours before an assessment of their mechanical and biochemical properties.

### Cell shortening and relengthening

The mechanical properties of cardiomyocytes were assessed using a SoftEdge MyoCam system (IonOptix Corporation, Milton, MA, USA) [5]. In brief, cells were placed in a Warner chamber mounted on the stage of an inverted microscope (Olympus, IX-70, Olympus Corporation, Tokyo, Japan) and superfused (approximately 1 mL/min at 25°C) with a buffer containing 131 mM NaCl, 4 mM KCl, 1 mM CaCl_2_, 1 mM MgCl_2_, 10 mM glucose and 10 mM 4-(2-hydroxyethyl)-1-piperazineethanesulfonic acid (HEPES), at pH 7.4. The cells were field-stimulated with a supra-threshold voltage at a frequency of 0.5 Hz for 3 ms using a pair of platinum wires placed on opposite sides of the chamber connected to a FHC stimulator (Brunswick, NE, USA). The studied myocyte was displayed on the computer monitor using an IonOptix MyoCam camera. IonOptix SoftEdge software was used to capture changes in cell length. Cell shortening and relengthening were assessed using the following indices: peak shortening (PS), the peak ventricular contractility; time-to-PS (TPS; contraction duration) and time-to-90% relengthening (TR_90_), the cardiomyocyte relaxation duration; and maximal velocities of shortening (+dL/dt) and relengthening (-dL/dt), the maximal velocities of ventricular pressure rise and fall.

### Intracellular Ca^2+ ^transient measurement

Myocytes were loaded with fura-2-acetoxymethyl ester (0.5 μM) for 10 minutes and fluorescence measurements were recorded with a dual-excitation fluorescence photomultiplier system (IonOptix). Cardiomyocytes were placed on an Olympus IX-70 inverted microscope and imaged through a Fluor × 40 oil objective. Cells were exposed to light emitted by a 75 W lamp and passed through either a 360 or a 380 nm filter, while being stimulated to contract at 0.5 Hz. Fluorescence emissions were detected between 480 and 520 nm by a photomultiplier tube after first illuminating the cells at 360 nm for 0.5 seconds then at 380 nm for the duration of the recording protocol (333 Hz sampling rate). The 360 nm excitation scan was repeated at the end of the protocol and qualitative changes in intracellular Ca^2+ ^concentration were inferred from the ratio of fura-2 fluorescence intensity (FFI) at the two wavelengths (360 and 380 nm). Fluorescence decay time was measured as an indication of the intracellular Ca^2+ ^clearing rate. Both single- and bi-exponential curve fit programs were applied to calculate the intracellular Ca^2+ ^decay constant [5].

### Histological examination

After anesthesia, hearts were excised and immediately placed in 10% neutral-buffered formalin at room temperature for 24 hours after a brief rinse with PBS. The specimens were embedded in paraffin, cut into 5 μm sections and stained with H & E as well as fluorescein isothiocyanate (FITC)-conjugated wheat germ agglutinin. Heart sections were stained with H & E for gross morphology analysis. Thereafter, the slides were washed three times with PBS, mounted with aqueous mounting media and cover-slipped. Cardiomyocyte cross-sectional areas were calculated on a digital microscope (× 400) using the Image J (version1.34S) software [5,20].

### Caspase-3 assay

Tissue homogenates were centrifuged (10,000 *g *at 4°C, 10 minutes) and pellets were lysed in an ice-cold cell lysis buffer. The assay was carried out in a 96-well plate with each well containing 30 μL cell lysate, 70 μL of assay buffer (50 mM HEPES, 0.1% 3-([3-cholamidopropyl]-dimethyllammonio)-1-propanesulfonate (CHAPS), 100 mM NaCl, 10 mM dithiothreitol and 1 mM ethylenediaminetetraacetic acid) and 20 μL of caspase-3 colorimetric substrate Ac-DEVD-pNA. The 96-well plate was incubated at 37°C for one hour, during which time the caspase in the sample was allowed to cleave the chromophore pNA from the substrate molecule. Caspase-3 activity was expressed as picomoles of pNA released per microgram of protein per minute [5].

### Aconitase activity

Mitochondrial aconitase, an iron-sulfur enzyme located in the citric acid cycle, is readily damaged by oxidative stress via removal of an iron from the [4Fe-4S] cluster. Mitochondrial fractions prepared from whole heart homogenate were resuspended in 0.2 mM sodium citrate. An aconitase activity assay (Aconitase Activity Assay Kit, Aconitase-340 Assay; OxisResearch, Portland, OR, USA) was performed according to the manufacturer instructions with minor modifications. Briefly, the mitochondrial sample (50 μL) was mixed in a 96-well plate with 50 μL trisodium citrate (substrate) in Tris-HCl pH 7.4, 50 μL isocitrate dehydrogenase (enzyme) in Tris-HCl, and 50 μL NADP in Tris-HCl. After incubating for 15 minutes at 37°C, the absorbance was dynamically recorded at 340 nm every minute for five minutes with a spectrophotometer. During the assay, citrate is isomerized by aconitase into isocitrate and eventually α-ketoglutarate. The Aconitase-340 Assay measures NADPH formation, a product of the oxidation of isocitrate to α-ketoglutarate. Tris-HCl buffer (pH 7.4) was served as the blank [25].

### Terminal deoxynucleotidyl transferase mediated dUTP nick end labeling assay

Terminal deoxynucleotidyl transferase mediated dUTP nick end labeling (TUNEL) staining of myonuclei positive for DNA strand breaks was determined using a fluorescence detection kit (Roche, Indianapolis, IN, USA) and fluorescence microscopy. Paraffin-embedded sections (5 μm) were incubated with Proteinase K solution for 30 minutes. TUNEL reaction mixture containing terminal deoxynucleotidyl transferase and fluorescein-dUTP was added to the sections in 50 μL drops and incubated for 60 minutes at 37°C in a humidified chamber in the dark. The sections were rinsed three times in PBS for five minutes each. Following embedding, sections were visualized with an Olympus BX-51 microscope equipped with an Olympus MaguaFire SP digital camera. DNase I and label solution were used as positive and negative controls. To determine the percentage of apoptotic cells, micrographs of TUNEL-positive and 4'-6-dia! midino-2-phenylindole-stained nuclei were captured using an Olympus fluorescence microscope and counted using the ImageJ software (ImageJ version 1.43r; National Institutes of Health) followed by manual exclusion of the false-positive staining from 10 random fields at 400 × magnification. At least 100 cells were counted in each field [26].

### Measurement of mitochondrial membrane potential

Murine cardiomyocytes were suspended in HEPES saline buffer and the mitochondrial membrane potential (ΔΨ_m_) was detected as previously described [27]. Briefly, after incubation with JC-1 (5 μM) for 10 minutes at 37°C, cells were rinsed twice by sedimentation using the HEPES saline buffer free of JC-1 before being examined under a confocal laser scanning microscope (Leica TCS SP2, Leica Microsystems Inc. Buffalo Grove, IL, USA) at an excitation wavelength of 490 nm. The emission of fluorescence was recorded at 530 nm (monomer form of JC-1, green) and at 590 nm (aggregate form of JC-1, red). Results in fluorescence intensity were expressed as the 590 nm to 530 nm emission ratio. The mitochondrial uncoupler carbonyl cyanide m-chlorophenylhydrazone (10 μM) was used as a positive control for the mitochondrial membrane potential measurement.

### Western blot analysis

The myocardial protein was prepared as previously described [27]. The antibodies used for western blotting included anti-PGC-1α, anti-UCP-2 (EMD Millipore Billerica, MA, USA), anti-ALDH2 (gift from Dr. Henry Weiner, Purdue University, West Lafayette, IN, USA), anti-GSK3β, anti-phosphorylated(p)-GSK3β (Ser^9^), anti-Akt, anti-pAkt (Thr^308^), anti-Foxo3a, anti-pFoxo3a (Thr^32^), anti-mTOR, anti-pmTOR (Ser^2448^), anti-PTEN, anti-pPTEN (Ser^380^), anti-sarcoendoplasmic reticulum Ca^2+^-ATPase (SERCA2a; Affinity Bioreagents Inc., Golden, CO, USA), anti-Na^+^-Ca^2+ ^exchanger (1:1000; Sigma, St. Louis, MO, USA), anti-phospholamban (1:500; Abcam, Cambridge, MA, USA) and anti-glyceraldehyde 3-phosphate dehydrogenase (GAPDH; loading control). Antibodies for GSK3β, pGSK3β, Akt, pAkt, Foxo3a, pFoxo3a, mTOR, pmTOR, PTEN and pPTEN were purchased from Cell Signaling Technology (Beverly, MA, USA) while antibody for PGC-1α was obtained from Santa Cruz Biotechnology (Santa Cruz, CA, USA) unless otherwise indicated. The membranes were incubated with horseradish peroxidase-coupled secondary antibodies. After immunoblotting, films were scanned and detected with a Bio-Rad Calibrated Densitometer Hercules, CA, USA)

### Data analysis

Data are presented as the mean ± standard error of the mean (SEM). Statistical comparison was performed by a one-way analysis of variance (ANOVA), with a two-way ANOVA for RER and physical activity studies, followed by Tukey's post hoc test. Significance was set as *P *< 0.05.

## Results

### General features, mitochondrial and metabolic properties of normal and diabetic mice

STZ treatment significantly reduced body but not organ weights in FVB and ALDH2 mice. Although STZ treatment did not affect the size of the kidney (organ-to-body weight ratio), it overtly increased heart and liver sizes in FVB but not ALDH2 mice. ALDH2 transgene did not affect the body and organ weights or organ sizes. As expected, blood glucose (fasting and postprandial) and free fatty acid levels were significantly elevated whereas plasma insulin levels were severely decreased in STZ-challenged mice compared with the non-diabetic FVB mice. ALDH2 did not affect the levels of fasting or postprandial blood glucose, serum free fatty acids or plasma insulin in either normal or diabetic groups (Table 1). Furthermore, experimental diabetes decreased both protein level and enzymatic activity of ALDH2, the effect of which was masked by ALDH2 overexpression. STZ elicited overt apoptosis (as evidenced by caspase-3 activity) and mitochondrial damage (reduced aconitase activity). Although ALDH2 enzymatic overexpression itself had little effect on apoptosis and mitochondrial function, it significantly attenuated or nullified diabetes-induced apoptosis and mitochondrial damage (Figure 1).

**Table 1:** Biometric parameters of control or diabetic FVB and ALDH2 mice

Parameter	FVB	FVB-STZ	ALDH2	ALDH2-STZ
Body weight (g)	30.3 ± 1.3	24.2 ± 0.7^a^	29.5 ± 1.1	26.1 ± 0.8^a^
Heart weight (mg)	165 ± 9	171 ± 8	163 ± 6	159 ± 5
Heart/body weight ratio (mg/g)	5.45 ± 0.19	7.23 ± 0.43^a^	5.66 ± 0.26	6.16 ± 0.18^b^
Liver weight (g)	1.54 ± 0.07	1.44 ± 0.07	1.52 ± 0.05	1.46 ± 0.06
Liver/body weight (mg/g)	51.2 ± 1.4	59.4 ± 2.3^a^	51.9 ± 1.9	54.9 ± 1.9
Kidney weight (g)	0.45 ± 0.03	0.39 ± 0.02	0.42 ± 0.02	0.40 ± 0.03
Kidney/body weight (mg/g)	14.8 ± 0.4	16.1 ± 0.8	14.4 ± 0.4	15.4 ± 0.8
Plasma insulin (ng/mL)	0.27 ± 0.03	0.05 ± 0.01^a^	0.28 ± 0.03	0.06 ± 0.02^a^
Fasting blood glucose (mM)	5.50 ± 0.26	19.7 ± 1.5^a^	5.43 ± 0.18	18.5 ± 1.7^a^
Postprandial blood glucose (mM)	9.94 ± 0.67	25.3 ± 1.5^a^	10.57 ± 0.54	26.5 ± 1.8^a^
Plasma free fatty acids (mM)	1.00 ± 0.11	1.30 ± 0.04^a^	1.00 ± 0.15	1.25 ± 0.08^a^

Mean ± SEM, n = 21 to 22 mice per group. ^a^*P *< 0.05 versus FVB group; ^b^*P *< 0.05 versus FVB-STZ group.

**Figure 1:** **Influence of streptozotocin and ALDH2 on expression and activity of ALDH2, apoptosis and mitochondrial function**. (**A) **ALDH2 expression; **(B) **ALDH2 enzymatic activity measured using spectrophotometry; **(C) **caspase-3 activity; **(D) **mitochondrial aconitase activity. Inset: Representative gel blots of ALDH2 and GAPDH (loading control) using specific antibodies. Mean ± SEM, n = 5 to 7 per group. *P < 0.05 versus FVB group; ^#^*P ***<**0.05 versus FVB-STZ group.

To evaluate the impact of ALDH2 overexpression on metabolic indices, calorimetric parameters were obtained in control and diabetic FVB and ALDH2 mice using the six-chamber Oxymax system (Columbus Instruments, Columbus, OH, USA) as previously described [19]. Diabetic FVB and ALDH2 mice had a significantly lower RER (VCO_2_/VO_2_), especially during the dark cycle, compared with control FVB and ALDH2 mice. This diabetes-associated change in RER was not due to altered physical activity. There was little difference in physical activity among the four mouse groups tested (Figure 2). These results indicate that STZ-induced diabetic mice oxidized a lower proportion of carbohydrate compared with control mice, reflecting a higher fractional reliance on lipid rather than glucose as the main energy source. ALDH2 overexpression did not alter the energy source globally in control or diabetic mice.

**Figure 2:** **Oxygen consumption and total activity during day and night time in FVB and ALDH2 transgenic mice treated with or without streptozotocin**. **(A) **Respiratory exchange ratio (RER) during day time; **(B) **RER at night; **(C) **total activity during day time; **(D) **total activity at night. Mean ± SEM, n = 4 to 5 mice per group. *P < 0.05 versus FVB group for both STZ groups.

### Echocardiographic properties of normal and diabetic mice

Heart rate and absolute LV mass (calculated using echocardiography) were comparable among all mouse groups, regardless of diabetic or ALDH2 state. However, diabetes increased the normalized LV mass value in the FVB but not ALDH2 group, consistent with its effect on gross heart weights. Experimental diabetes significantly increased EDD and ESD and decreased wall thickness, the effect of which was mitigated by ALDH2. Interestingly, STZ treatment significantly depressed fractional shortening in FVB mice. ALDH2 mitigated the diabetes-induced decrease in fractional shortening without eliciting any effect itself (Figure 3).

**Figure 3:** **Echocardiographic properties in FVB and ALDH2 transgenic mice treated with or without streptozotocin**. **(A) **Representative echocardiographic images; **(B) **heart rate; **(C) **wall thickness; **(D) **left ventricular (LV) end-diastolic diameter; **(E) **LV end-systolic diameter; **(F) **LV mass; **(G) **LV mass normalized to body weight; **(H) **fractional shortening. Mean ± SEM, n = 12 to 13 mice per group. *P **<**0.05 versus FVB group; ^#^*P ***<**0.05 versus FVB-STZ group.

### Cardiomyocyte contractile and intracellular Ca^2+ ^properties

Neither experimental diabetes nor ALDH2 overexpression affected resting cell length, as depicted in Figure 4. Experimental diabetes significantly reduced PS and maximal velocity of shortening and relengthening (± dL/dt) as well as prolonged TPS and TR_90 _in FVB cardiomyocytes, reminiscent of our earlier findings [28,29]. Importantly, ALDH2 abolished diabetes-induced mechanical abnormalities without eliciting any notable effect by itself. To explore the potential mechanism of action involved in the ALDH2-elicited beneficial effects against experimental diabetes, fura-2 fluorescence microscopy was employed to monitor the intracellular Ca^2+ ^homeostasis. Data presented in Figure 5 reveal a significantly depressed intracellular Ca^2+ ^rise in response to electrical stimulus (ΔFFI) and reduced intracellular Ca^2+ ^decay rate (single or bi-exponential curve fit) along with unchanged baseline intracellular Ca^2+ ^in cardiomyocytes from STZ-treated mouse hearts. ALDH2 overexpression negated STZ-induced prolongation in intracellular Ca^2+ ^decay and depression in ΔFFI with little effect on baseline FFI. Last but not least, the ALDH2 transgene itself did not affect the intracellular Ca^2+ ^indices tested.

**Figure 4:** **Cardiomyocyte contractile properties in FVB and ALDH2 transgenic mice treated with or without streptozotocin**. **(A) **Resting cell length; **(B) **peak shortening (PS), normalized to cell length; **(C) **maximal velocity of shortening (+ dL/dt); **(D) **maximal velocity of relengthening (- dL/dt); **(E) **time-to PS (TPS); **(F) **time-to-90% relengthening (TR_90_). Mean ± SEM, n = 101 to 102 cells from four mice per group. *P **<**0.05 versus FVB group; ^#^*P ***<**0.05 versus FVB-STZ group.

**Figure 5:** **Cardiomyocyte intracellular Ca^2+ ^handling properties in FVB and ALDH2 transgenic mice treated with or without streptozotocin**. **(A) **Resting fura-2 fluorescence intensity (FFI); **(B) **electrically-stimulated rise in FFI (ΔFFI); **(C) **intracellular Ca^2+ ^decay rate (single exponential); **(D) **intracellular Ca^2+ ^decay rate (bi-exponential). Mean ± SEM, n = 76 to 77 cells from four mice per group. *P **<**0.05 versus FVB group; ^#^*P <*0.05 versus FVB-STZ group.

### Effect of ALDH2 on diabetes-induced change in myocardial histology

To assess the impact of ALDH2 overexpression on myocardial histology after STZ treatment, heart gross morphology and the cardiomyocyte cross-sectional area were examined. Low magnification transverse heart sections indicated reduced LV wall thickness and enlarged chamber size in mice with experimental diabetes, with lesser alteration in ALDH2 transgenic mice. Findings from FITC-conjugated wheat germ staining sections revealed increased cardiomyocyte area after the induction of experimental diabetes, consistent with increased normalized LV mass, EDD and ESD in FVB-STZ mice. The experimental diabetes-induced change in cardiomyocyte size was effectively ablated by ALDH2 overexpression while the ALDH2 transgene itself did not affect cardiomyocyte size (Figure 6).

**Figure 6:** **Histological analyses in hearts from FVB and ALDH2 transgenic mice treated with or without streptozotocin**. **(A-D) **Representative photomicrographs from gross morphological view of transverse myocardial sections (scale bar = 1 mm). **(E-H) **Representative fluorescein isothiocyanate-conjugated wheat germ agglutinin staining depicting cardiomyocyte size (× 200; scale bar = 100 μm). **(I) **Quantitative cardiomyocyte cross-sectional (transverse) area from 60 cells from three mice per group. Mean ± SEM, *P < 0.05 versus FVB; ^#^*P *< 0.05 versus FVB-STZ group.

### Effects of ALDH2 on diabetes-induced apoptosis and mitochondrial damage

To further examine the mechanism(s) of action behind ALDH2-elicited protection against STZ-induced cardiac mechanical dysfunction, the myocardium and cardiomyocytes from normal or diabetic FVB and ALDH2 mice were examined for myocardial apoptosis, using TUNEL staining, and mitochondrial integrity, using JC-1 fluorescence microscopy. Results shown in Figure 7 (panels A-I) indicate that the TUNEL-positive cells were more abundant in STZ-treated FVB mice, the effect of which was significantly attenuated by ALDH2 overexpression. ALDH2 itself did not affect myocardial apoptosis. Our fluorescence data displayed in Figure 7 (panels J and K) revealed loss of mitochondrial membrane potential in cardiomyocytes from STZ-treated FVB mice, the effect of which was reconciled by ALDH2 overexpression. ALDH2 itself did not affect the mitochondrial membrane potential. These findings indicate a corroborative role of apoptosis and mitochondrial function in ALDH2-offered cardioprotection against experimental diabetes.

**Figure 7:** **Effect of streptozotocin and ALDH2 on myocardial apoptosis and mitochondrial membrane potential using TUNEL staining and JC-1 fluorescence**. TUNEL-positive nuclei were visualized with fluorescein (green) in panels **(A) **FVB, **(C) **FVB-STZ, **(E) **ALDH2 and **(G) **ALDH2-STZ. All nuclei were stained with 4'-6-diamidino-2-phenylindole (blue) in panels **(B) **FVB, **(D) **FVB-STZ, **(F) **ALDH2 and **(H) **ALDH2-STZ. Original magnification × 400. **(I) **Quantified data. **(J) **Quantitative analysis of cardiomyocyte mitochondrial membrane potential using JC-1 ratio in FVB and ALDH2 mice treated with or without STZ (10 μM carbonyl cyanide m-chlorophenylhydrazone was used as a positive control). **(K) **Representative JC-1 fluorochrome images depicting mitochondrial membrane potential in cardiomyocytes. Mean ± SEM, n = 12 and 7 fields from three mice per group for panel I and J, respectively. *P < 0.05 versus FVB group; ^#^*P *< 0.05 versus FVB-STZ group.

### Expression of UCP-2, PGC1α, SERCA2a, Na^+^-Ca^2+ ^exchanger and phospholamban

To explore the possible mechanism behind ALDH2 and diabetes-induced responses on cardiac function, particularly on mitochondrial function and intracellular Ca^2+ ^homeostasis, western blot analysis was performed to assess the levels of the key mitochondrial proteins UCP-2 and PGC1α as well as the essential intracellular Ca^2+ ^regulatory proteins SERCA2a, Na^+^-Ca^2+ ^exchanger and phospholamban. Our data shown in Figure 8 depict that diabetes significantly downregulated the expression of UCP-2, PGC1α, SERCA2a and Na^+^-Ca^2+ ^exchanger while upregulating the level of phospholamban in FVB mice. Although the ALDH2 transgene itself did not alter the expression of UCP-2, PGC1α, SERCA2a, Na^+^-Ca^2+ ^exchanger or phospholamban, it nullified STZ-induced changes in all five.

**Figure 8:** **Western blot analysis of the mitochondrial proteins UCP-2 and PGC1α as well as the Ca^2+ ^regulatory proteins SERCA2a, Na^+^-Ca^2+ ^exchanger and phospholamban in myocardium from FVB and ALDH2 mice treated with or without streptozotocin**. **(A) **Representative gel blots of UCP-2, PGC1α, SERCA2a, Na^+^-Ca^2+ ^exchanger, phospholamban and GAPDH (loading control) using specific antibodies; **(B) **UCP-2; **(C) **PGC1α; **(D) **SERCA2a; **(E) **Na^+^-Ca^2+ ^exchanger; **(F) **phospholamban. All proteins were normalized to the loading control GAPDH. Mean ± SEM, n = 5 to 6 mice per group. *P < 0.05 versus FVB group; ^#^*P *< 0.05 versus FVB-STZ group.

### Western blot analysis for Akt, GSK3β, Foxo3a, mTOR and PTEN signaling

To examine possible signaling mechanism(s) involved in the ALDH2-offered protection against diabetes-induced myocardial anomalies, the expression and phosphorylation of post-insulin receptor signaling, including Akt and the Akt downstream signaling molecules GSK3β, Foxo3a and mTOR, were evaluated. Western blot findings revealed that diabetes overtly dampened phosphorylation of Akt, GSK3β and Foxo3a without affecting that of mTOR, the effect of which was mitigated by ALDH2 overexpression. Neither diabetes nor ALDH2 affected the pan protein expression of Akt, Foxo3a or mTOR (Figure 9). To explore the possible mechanisms responsible for ALDH2- and experimental diabetes-elicited changes in Akt phosphorylation, levels of pan and pPTEN, a negative regulator of Akt signaling, were examined in control and diabetic FVB and ALDH2 mice. Our data shown in Figure 10 revealed that STZ treatment significantly increased phosphorylation of PTEN (both absolute and normalized value) without affecting pan protein expression of PTEN, the effect of which was mitigated by ALDH2 overexpression. The ALDH2 transgene itself did not affect pan or phosphorylated levels of PTEN.

**Figure 9:** **Phosphorylation of Akt, GSK3β, mTOR and Foxo3a in myocardium from FVB and ALDH2 mice treated with or without streptozotocin**. **(A) **pAkt-to-Akt ratio; **(B) **pGSK3β-to-GSK3β ratio; **(C) **pmTOR-to-mTOR ratio; **(D) **pFoxo3a-to-Foxo3a ratio. Insets: representative gel blots of pan and phosphorylated Akt, GSK3β, mTOR and Foxo3a (GAPDH as loading control) using specific antibodies. Mean ± SEM, n = 6 to 7 mice per group. *P < 0.05 versus FVB group; ^#^*P *< 0.05 versus FVB-STZ group.

**Figure 10:** **Total and phosphorylated PTEN in myocardium from FVB and ALDH2 mice treated with or without streptozotocin**. **(A) **Representative gel blots of pan and phosphorylated PTEN and GAPDH (used as loading control) using specific antibodies; **(B) **pan PTEN expression; **(C) **pPTEN levels; **(D) **pPTEN-to-PTEN ratio. Mean ± SEM, n = 6 mice per group. *P < 0.05 versus FVB group; ^#^*P *< 0.05 versus FVB-STZ group.

### Influence of ALDH2 activation, mitochondrial uncoupling and GSK3β inhibition on high glucose-induced cardiomyocyte mitochondrial and contractile responses

To further examine the causal relationships between ALDH2-induced mechanical and mitochondrial responses in diabetes, cardiomyocytes from control FVB mice were exposed to high glucose (25.5 mM) in the absence or presence of the ALDH2 activator Alda-1 (20 μM), the mitochondrial uncoupler FCCP (1 μM) or the GSK3β inhibitor SB216763 (10 μM) for 12 hours [6,9,30] prior to an assessment of mechanical and biochemical properties. Figure 11 depicts that high glucose significantly dampened mitochondrial function (shown as loss of aconitase activity) and cardiomyocyte contractile function (shown as reduced PS, ± dL/dt and prolonged TR_90_), the effect of which was abolished by Alda-1 and SB216763, without any additive effect between the two. Interestingly, FCCP abolished Alda-1-induced beneficial mitochondrial and mechanical effects. There was little effect on mitochondrial integrity and mechanical function by the pharmacological inhibitors themselves (data not shown for FCCP).

**Figure 11:** **Influence of the ALDH2 agonist Alda-1 on high glucose-induced responses of aconitase activity and cardiomyocyte contractile properties**. Cardiomyocytes from control FVB mice were exposed to high glucose (HG; 30 mM) in the absence or presence of Alda-1 (20 μM), the mitochondrial uncoupler FCCP (1 μM) or the GSK3β inhibitor SB216763 (10 μM) for 12 hours prior to assessment of mitochondrial and mechanical properties. **(A) **Aconitase activity; **(B) **peak shortening (PS; normalized to cell length); **(C) **maximal velocity of shortening (+ dL/dt); **(D) **maximal velocity of relengthening (- dL/dt); **(E) **time-to PS (TPS); **(F) **time-to-90% relengthening (TR_90_). Mean ± SEM, n = 5 isolations (panel A) or 72 to 73 cells per group (Panel B-F). *P < 0.05 versus control group; ^#^*P *< 0.05 versus HG group.

## Discussion

Earlier findings from our group indicated that ALDH2 may rescue against ischemic and alcoholic injuries to the heart [3,7,15]. Data from this study provides, for the first time, compelling evidence that ALDH2 protects against diabetes-induced myocardial remodeling and contractile defect through lessened apoptosis, preserved mitochondrial function and post-insulin receptor signaling, including phosphorylation of Akt, GSK3β and Foxo3a transcriptional factor. These data favor a likely role of the activation of Akt and GSK3β as well as inactivation (phosphorylation) of Foxo3a in ALDH2-elicited preservation of mitochondrial and mechanical function in diabetes. Our data further reveal that ALDH2 may preserve Akt activation in diabetes through ablation of diabetes-induced mitochondrial injury and/or increasing the phosphorylation of PTEN, a negative regulator of Akt [16]. An analysis of global metabolism indicated that ALDH2 failed to alter diabetes-induced changes in plasma levels of glucose (fasting and postprandial), insulin and serum free fatty acids, the RER or total physical activity, excluding the possibility of a potential cardiac protective effect secondary to any ALDH2-elicited global metabolic benefits. Taken together, these findings should lead to a better understanding of the role of ALDH2 in myocardial anomalies in diabetes.

Reduced contractility and prolonged duration of systole as well as diastole are hallmarks of diabetic cardiomyopathy [17,28,29]. Findings from our present study revealed reduced fractional shortening; enlarged EDD and ESD; decreased wall thickness, PS and ± dL/dt; and prolonged TPS and TR_90 _in whole hearts and isolated cardiomyocytes in diabetic mice. These findings are similar to our previous findings [17,28,29]. Several mechanisms may be postulated for diabetes-related abnormalities such as impaired intracellular Ca^2+ ^homeostasis and oxidative stress [28,29]. In our study, the impaired intracellular Ca^2+ ^handling (reduced intracellular Ca^2+ ^clearance and intracellular Ca^2+ ^rise (ΔFFI)) may likely underscore the prolonged duration of contraction and relaxation and the reduced PS, maximal velocity of shortening and relengthening and fractional shortening observed in STZ-induced diabetic mouse hearts. The fact that the ALDH2 transgene reconciled STZ-induced intracellular Ca^2+ ^mishandling favors a possible role of intracellular Ca^2+ ^homeostasis in diabetes-induced myocardial dysfunction and ALDH2-offered protection, somewhat reminiscent of the beneficial role of mitochondrial protection against diabetes or obesity-induced myocardial dysfunction [31,32]. Our findings revealed a loss of mitochondrial membrane potential and overt apoptosis (demonstrated by caspase-3 and TUNEL) along with downregulated levels of PGC1α and UCP-2 in STZ-induced diabetic hearts, suggesting a corroborative role of mitochondrial dysfunction and apoptosis in diabetic cardiomyopathy, as reported previously [31]. In addition, our observations that the ALDH2 transgene restored downregulated expression of SERCA2a and Na^+^-Ca^2+ ^exchanger as well as upregulated phospholamban in diabetes also support a role of intracellular Ca^2+ ^homeostasis in diabetes-induced cardiac contractile dysfunction and ALDH2-offered protection.

Perhaps our most significant finding is that ALDH2 overexpression reconciled diabetes-induced cardiac remodeling (represented by cardiomyocyte cross-sectional area, changes in LV wall thickness, ESD and EDD) and contractile dysfunction in association with preserved myocyte survival and mitochondrial integrity. These beneficial effects of ALDH2 in cardiac geometry and function, cell survival and mitochondrial integrity were seen despite the persistent hyperglycemic and hyperlipidemic environments in STZ-induced experimental diabetes, thus excluding a possible secondary effect for ALDH2-induced protection against diabetic cardiomyopathy. This is further supported by the fact that ALDH2 failed to alter global metabolism (RER and physical activity) in diabetes. In our study, STZ failed to elicit any hypertrophic effect as evidenced by absolute heart weight and LV mass, although it enhanced cardiomyocyte size and heart-to-body weight ratio, and normalized LV mass. These effects were likely due to an STZ-induced loss in body weight. Interestingly, ALDH2 overexpression attenuated diabetes-induced changes in cardiomyocyte, heart and LV sizes, possibly due to the antagonism of ALDH2 against diabetes-induced cardiac apoptosis and mitochondrial damage. Both apoptosis and mitochondrial damage are known to regulate cardiac remodeling in diabetes and obesity [31,33]. Our observation of preserved levels of the mitochondrial proteins PGC1α and UCP-2 as well as of aconitase activity and mitochondrial membrane potential in ALDH2 mice after STZ treatment strongly supported a role of mitochondrial function in ALDH2-offered cardioprotection. The therapeutic role of the mitochondrial protein ALDH2 in diabetes is consistent with the fact that the protein level and enzymatic activity of ALDH2 are both reduced in experimental diabetes [13] (also seen in our study) while inactive ALDH2 promotes hyperglycemia and enhances the risk of diabetes [14].

It is noteworthy that the reduction in the ALDH2 expression and activity is relatively minor although such subtle loss of ALDH2 may be sufficient to trigger overt changes in mitochondrial integrity and cell survival. Although it is beyond the scope of our current study, the main substrate for ALDH2 detoxification, aldehydes, serve as the main source for oxidative stress and pathological changes in disease condition. Even with a moderately reduced ALDH2 level, sublethal levels of aldehydes may accumulate and interact with functional signaling systems to impose oxidative damage and associated gene alterations in response to the stress challenge [34]. The notion that ALDH2 protects against diabetic cardiomyopathy through preservation of mitochondrial integrity was further substantiated by our *in vitro *findings. Our results revealed that the ALDH2 activator Alda-1 effectively rescued against high glucose-induced mitochondrial and mechanical dysfunctions, and this effect was nullified by the mitochondrial uncoupling compound FCCP. These data convincingly support the permissive role of mitochondria in ALDH2-offered cardioprotection against hyperglycemia-induced anomalies.

Data from our study showed dampened phosphorylation of the post-insulin receptor signaling Akt, GSK3β and Foxo3a in STZ-treated diabetic hearts, in line with mitochondrial injury in diabetes and observations from our earlier studies [28,35]. These signaling molecules play an essential role in the maintenance of cardiac survival, structure and function. Akt, GSK3β and mTOR are essential post-insulin receptor signaling molecules, which may be compromised after mitochondrial injury and contribute to apoptosis and cardiac dysfunction in pathological conditions [10,14,36]. Our data revealed that diabetes dampened phosphorylation of Akt and its downstream signaling molecules Foxo3a and GSK3β (although not mTOR), the effect of which was nullified by ALDH2 transgene. The decrease in the phosphorylation of Foxo3a and GSK3β is expected to result from dampened Akt phosphorylation. The reduced phosphorylation of Foxo3a appears to coincide with overt mitochondrial injury (as evidenced by mitochondrial membrane potential and levels of PGC1α, UCP-2 and aconitase) and apoptosis (demonstrated by caspase-3 and TUNEL staining) after STZ treatment, as reported previously by our group using the same diabetic model [35]. GSK3β, a serine/threonine kinase downstream of Akt that is inactivated by oxidative stress through the phosphorylation of Ser9, serves as a negative regulator of cardiac hypertrophy and mitochondrial function through mitochondrial permeation pore opening [24,25,37]. Data from our study revealed that ALDH2 abrogated the diabetes-induced decrease in GSK3β phosphorylation, aconitase activity and levels of PGC1α and UCP-2, favoring a possible role of GSK3β signaling and mitochondrial protection in ALDH2-offered cardioprotection. This is supported by the finding that GSK3β inhibition using SB216763 and mitochondrial uncoupling using FCCP respectively ablated high glucose and Alda-1-induced mitochondrial and mechanical changes.

Mitochondrial injury is known to compromise insulin signaling at both insulin receptor and post-receptor levels [30]. A recent report from our group revealed that protection of mitochondrial integrity using cardiac-specific overexpression of insulin-like growth factor 1 effectively alleviates high fat diet intake-induced loss of insulin sensitivity, oxidative stress and contractile dysfunction in the heart [38], supporting the pivotal role of mitochondria in the maintenance of cardiac insulin signaling. Nonetheless, our data also depicted elevated phosphorylation of the Akt negative regulator PTEN in experimental diabetes, the effect of which was mitigated by ALDH2. This finding favors a possible role for PTEN in ALDH2 overexpression-rescued Akt activation in experimental diabetes. These observations suggest that ALDH2 offers cardioprotection against experimental diabetes, possibly through suppressed PTEN phosphorylation and subsequently preserved Akt-GSK3β phosphorylation, leading to protected mitochondrial integrity.

## Conclusion

In summary, findings from our present study reveal a role of ALDH2 in the protection against diabetic cardiomyopathy, possibly via an Akt-GSK3β-mediated preservation of cell survival and mitochondrial integrity. These data indicate not only a role of ALDH2 in the prevalence of diabetic cardiomyopathy but also some therapeutic promise for ALDH2 in the management of diabetic complications. As the important cardioprotective aspects of ALDH2 begin to be unveiled, clinical implications of ALDH2, in particular ALDH2 polymorphism, still remain to be explored. Further studies should focus on a better elucidation of the link between the ALDH2 gene and cardiovascular risk in diabetic populations.

## Abbreviations

+ dL/dt: maximal velocity of shortening; - dL/dt: maximal velocity of relengthening; ALDH2: mitochondrial aldehyde dehydrogenase; ANOVA: analysis of variance; EDD: end-diastolic diameter; ELISA: enzyme-linked immunosorbent assay; ESD: end-systolic diameter; FCCP: carbonyl cyanide 4-trifluoromethoxyphenylhydrazone; FFI: fura-2 fluorescence intensity; FITC: fluorescein isothiocyanate; GADPH: glyceraldehyde 3-phosphate dehydrogenase; GSK3β: glycogen synthase kinase-3β; H & E: hematoxylin and eosin stain; HEPES: 4-(2-hydroxyethyl)-1-piperazineethanesulfonic acid; LV: left ventricular; mTOR: mammalian target of rapamycin; p: phosphorylated; PBS: phosphate-buffered saline; PPAR: peroxisome proliferator-activated receptor; PTEN: phosphatase and tensin homologue on chromosome ten; PS: peak shortening; RER: respiratory exchange ratio; SEM: standard error of the mean; SERCA2a: sarcoendoplasmic reticulum Ca2+-ATPase; STZ: streptozotocin; TPS: time-to peak shortening; TR_90_: time-to-90% relengthening; TUNEL: terminal deoxynucleotidyl transferase mediated dUTP nick end labeling assay.

## Competing interests

The authors declare that they have no competing interests.

## Authors' contributions

YZ, SAB, NH and JRM participated in data collection; YZ, HW, JR designed the study, secured the research funding and wrote the manuscript. All authors have read and approved the final manuscript.

## Pre-publication history

The pre-publication history for this paper can be accessed here:

http://www.biomedcentral.com/1741-7015/10/40/prepub
